RETRACTED

# Probabilistic Statistics-Based Endurance Life Prediction of Bridge Structures

**DOI:** 10.1155/2022/8035028

**Published:** 2022-06-15

**Authors:** Yanan Zhang

**Affiliations:** School of Mathematics and Computer Science, Shaanxi University of Technology, Hanzhong 723001, China

## Abstract

With the massive construction of bridge infrastructures, bridge health monitoring systems have gradually matured in application and research, but previous research has primarily focused on structural damage detection and bridge safety warnings based on valid data. The structural details of steel bridge panels and structural systems are determined by the coupling effects of many intrinsic and extrinsic uncertainties, such as material properties, structural characteristics, manufacturing processes, and random traffic loads. The evaluation of fatigue is a difficult task. This article first builds a big data platform, utilizing its high-efficiency parallel computing capability and highly fault-tolerant distributed file system to achieve second-level monitoring data processing; ensuring real-time data cleaning, data analysis, and safety warning; and building a big data analysis and processing platform with high reliability, high availability, high storage efficiency, and high scalability of bridge health monitoring. The big data platform chooses HDFS for offline data storage and Spark for data analysis and modelling after comparing and analysing the benefits and drawbacks of various big data technologies. Kafka is used for caching real-time data, and Spark-streaming is used for reading data and real-time processing. Finally, the platform's superiority and reliability in terms of offline computing performance, real-time online performance, scalability, and fault tolerance are confirmed through experimental analysis; the optimal data cleaning method is derived by comparing and analysing monitoring data noise, jump point, and drift phenomena. This part of the research is based on bridge temperature data with stable signals and bridge strain data with fluctuating signals, taking into account the influence of different data types; the corresponding data missing repair algorithms are proposed for different types of data to form a complete and general data patching method process. The probabilistic fracture mechanics theory, in comparison to the traditional deterministic fatigue assessment method, can better reflect the essential uncertainty of fatigue problems and is an effective way to assess the fatigue performance of orthotropic steel bridge decks. The goal of data patching is to ensure data recovery accuracy of over 90%, with no patching repair required for monitoring data with too much missing data. The endurance life of bridge structures is predicted using a big data probabilistic statistics approach based on a variety of factors such as material properties, construction characteristics, manufacturing processes, and random traffic loads.

RETRACTED

## 1. Introduction

Bridges are the key nodes in the traffic lifeline project, and also show the strength of the country in social and economic development. In recent times, as the number of bridges increases and the age of bridges increases, the focus of bridgework is changing from “reconstruction rather than maintenance” to “construction and maintenance,” and even “management and maintenance.” However, compared with the breakthrough achievements in the fields of super flexible structure analysis, deep-water foundation design and construction, and super span bridge construction, there is a serious lack of research in bridge maintenance technology, and a weak reserve of bridge safety and health technology, resulting in the structural performance of bridges decaying before they get old, and the service life is generally much lower than the design life, and even safety accidents occur frequently. According to statistics, 60% of the actual life of the bridge is less than 25 years, nearly 800,000 highway bridges, the proportion of dangerous bridges is close to 15%, and the hidden danger is huge.

Large steel bridges are critical nodes and hubs in road traffic engineering, and orthotropic anisotropic steel bridge deck panels as the preferred deck structure for their main girders are required to ensure their safety and reliability in high-quality service during the design life. The fatigue cracking problem and secondary diseases such as deck pavement damage caused by the coupling influence of multiple factors such as structural characteristics and force system, material properties, environmental effects, and construction quality run through the entire process of application and development of orthotropic steel bridge panels, according to engineering application practice and research at home and abroad. It is difficult to repair and raise the overall cost of ownership, making it a management issue and a technical bottleneck that stymies the long-term development of steel bridges.

After large-scale new construction, developed countries have shifted their focus to the repair, reinforcement, and renovation of old buildings, and reconstruction is not only less expensive than new construction but also recovers the investment faster. Because of the current state of bridges, infrastructure investments should be directed toward the expansion and reconstruction of old and dangerous bridges. Durability assessment and life prediction are needed to develop scientifically developed repair, strengthening, and renovation plans for existing service structures. On the one hand, durability assessment and service life prediction can reveal the structure's potential hazards, and based on the results, the structure can be repaired and strengthened at an early stage of structural performance degradation, extending the structure's service life, reducing economic loss, and mitigating the serious energy and environmental problems caused by durability failure. On the other hand, it can reveal internal and external factors that affect the structure's life span. The existing deterministic methods are difficult to accurately consider the influence of the random characteristics of the abovementioned key factors and may obtain unsafe fatigue performance evaluation results. Aiming at the shortcomings of the existing deterministic evaluation methods, this article conducts systematic research on key issues such as fatigue load, crack growth, and fatigue reliability model and introduces the theory of random process and elastic-plastic fracture mechanics respectively to explore the effect of constant amplitude and random load. Based on the fatigue crack propagation characteristics, the probability and statistics theory and reliability theory are unified into the fatigue evaluation framework based on fracture mechanics, and a fatigue reliability evaluation method based on probabilistic fracture mechanics is proposed. Thus, targeted investments can be made according to the surrounding environment, usage, economic conditions, etc., which helps to improve the design level and construction quality of the project and improve the theory and method of new structural durability design.

RETRACTED

## 2. Related Works

The research results of bridge health monitoring are becoming more mature, and some large bridges in the United States and abroad are equipped with various monitoring instruments and monitoring devices, as shown in Figure 1 for factors affecting bridge endurance life, primarily to monitor these factors. The first health monitoring systems were installed and researched in foreign countries in 1922 on the Ironton-Russell suspension bridge in the United States, which had undergone several repairs and reinforcements, so the relevant units installed health monitoring systems to monitor the stress changes of the bridge structure, and the bridge was operated safely for the next decades until it was demolished [1]. In addition to the installation of bridge health monitoring, research in the field of health monitoring has tended to be rich and mature, and bridge health monitoring has evolved in the direction of intelligence and digitalization in the current era of big data.

RETRACTED

The material fracture prediction is closely related to the material type, chemical composition, and manufacturing process, and its magnitude is the key factor determining the fatigue crack propagation characteristics of the structural details of the steel bridge deck. The fracture parameter values of different steels are quite different and show significant random characteristics due to the influence of the inhomogeneity of the material microstructure. In foreign studies, literature [2] designed a bridge health monitoring system based on strain monitoring data, using the strain monitoring data collected to determine the stresses generated by live loads, to identify valuable parameters such as live load distribution factors and peaks, and to evaluate the structural health state of the bridge. Literature [3] investigated the improvement in the existing bridge monitoring system and proposed a method for information integration. The method uses a Bayesian probability model to obtain data and information from the structural health monitoring system to predict the probability of extreme values generation. This bridge health monitoring system has been applied to bridges in Wisconsin with good results. A method for adaptive identification of truss structures based on the Lyapunov method is proposed in the literature [4]. The Lyapunov method provides guaranteed convergence for parameter estimation in the identification. The finite element analysis method is used to identify the simulation model. The simulation results show that the adaptive estimation method can track the changes over time, thus providing monitoring of the degraded structure. Literature [5] utilized an enhanced structural health monitoring system using stream processing and artificial neural network techniques (SPAN Net) and applied it to a bridge in Bangkok. The system provides real-time monitoring and early warning mechanisms for bridge structures by applying wireless sensor networks, real-time data stream processing, and weighted attack maps based on measured bending strains.

Although Chinese bridge monitoring research is lagging behind that of other countries, bridge health monitoring researchers have conducted scientific research on health monitoring systems and practical research on various major bridge structures in China. Bridge health monitoring combined with machine learning and big data platforms are gradually emerging in today's wave of big data and artificial intelligence. Literature [6] proposed a method to evaluate the service status of bridge structures using a five-layer deep learning network and built an accurate finite element model of bridge structures based on bridge monitoring data. The pattern classification technique using neural networks was analysed using dynamic networks and genetic algorithms in literature [7], and its effectiveness in identifying structural damage of bridges was analysed in real tests, demonstrating the technique's feasibility. Literature [8] used radial basis function (RBF) neural networks to identify bridge damage and established guidelines for locating judged damage as well as an evaluation method for the identification effect. Literature [9] looked into a two-step method for damage detection based on a generalized regression neural network (GRNN), which is a variant of the radial basis (RBF) network with a faster training speed and a stronger nonlinear mapping capability, and network training can be completed instantly with high fitting accuracy. However, only a few typical simple bridge structures have been numerically simulated in the experimental validation stage, and there is still a significant gap in applying it to the damage identification of large bridge structures. The Korhonen clustering network was used in literature [10] to analyse isolated points of bridge monitoring data, as well as the analysis and early warning reference of bridge structure abnormalities based on this; the a priori model for bridge condition assessment was also established to explore the potential association rules among the attributes of bridge data, providing a data-supported basis for bridge condition assessment.

RETRACTED

## 3. A Probabilistic Statistics-Based Approach to Bridge Life Prediction

### 3.1. Bridge Structure Durability Life Prediction Method

The service life of bridge structures has certain uncertainty due to the environment they are in and the level of corrosion stress. However, how to accurately predict the reliability of bridge structures during service; guide, overhaul, and improve their reliability; and ensure their service life under harsh environments is a concern for bridge durability researchers [11]. The establishment of a reliable theoretical relationship between the durability deterioration process and time, based on which the service life of bridge structures can be assessed qualitatively and quantitatively, is referred to as life prediction of bridge structures. Empirical prediction, comparative performance prediction, accelerated test prediction, mathematical model prediction, and probabilistic analysis (stochastic process) prediction are the main methods for life prediction of bridge structures in general, and these methods are often used interchangeably in practice, rather than just one. Due to the drawbacks of empirical and performance comparison prediction methods [12], such as low prediction reliability, large errors, and significant limitations in the application of new materials, three bridge structure durability prediction methods are widely used.

RETRACTED

#### 3.1.1. Accelerated Test Prediction Method

Accelerated testing is based on test simulations to increase the level of corrosion stress, such as increasing the temperature, humidity, and concentration of corrosive ions, to accelerate the deterioration process of bridge structure durability and shorten its actual service life. This method can predict the service life of reinforced concrete very well if the acceleration mechanism is reasonably designed, the test operation is reasonable, and the data collection method is correct [13]. But often in practice, due to the acceleration test mechanism and corrosion stress level and the actual engineering corrosion stress in the process of durable deterioration of reinforced concrete between the match to be clear, whether too high or too low scholars question the attitude, that is, the precise value of the acceleration factor (K) has ambiguity. According to the fatigue damage characteristics of orthotropic steel bridge decks, the effects of key factors such as materials, loads, and defects are comprehensively considered, and the fatigue reliability and time-varying laws of typical structural details during service as well as fatigue crack propagation characteristics are reasonably predicted. The evaluation method of the orthotropic steel bridge deck is the primary issue in fatigue evaluation.  Figure 2 shows the accelerated experimental prediction method process.

#### 3.1.2. Mathematical Model Prediction Method

The mathematical model prediction method is the most widely used in today's study of bridge structure life prediction, and it is primarily based on the steel corrosion model, which is embodied primarily through the carbonation and chloride ion diffusion theory and other calculation models, and it has now become an important life prediction tool. The accuracy and reliability of life prediction, on the other hand, are closely linked to the logic of mathematical models, the selection of material-related parameters, and the compatibility of environmental factors, and the results are somewhat absolute.

#### 3.1.3. Probabilistic Analysis and Prediction Method

The probabilistic analysis prediction method expresses the relationship between the service life of bridge structures and time through the function of development evolution, and the prediction result is the non-mean service life (deterministic model), but the service life with a stochastic process, that is, the probability that the durability of bridge structures will fail at a certain service time point. The durability degradation of bridge structures is a changing process during the service life of bridge structures because it is the result of the coupling of various factors. For example, the hydration of MgSO_4_ and cementitious materials has a double effect on bridge durability degradation. According to the need for durability assessment, the environment in which the structure is located should be investigated. Temperature, humidity, aggressive material gases, liquids and solids, freeze-thaw cycles and scouring, wear and tear, and other factors are all taken into account. The corresponding original design data and the survey of the completed acceptance data should both be completed at the same time. Meanwhile, the initial durability of the bridge structure is a continuous strengthening process with the addition of admixtures and dopants, and given this, the probabilistic analysis-based method of predicting the life of bridge structures is more reasonable than other methods. Furthermore, the service life prediction based on a deterministic model has certain ambiguity in the process of bridge structure life prediction, so it is necessary to use a probabilistic method to predict its service life. The probabilistic analysis prediction method is depicted in Figure 3.

RETRACTED

The durability of bridge structures has always been the focus of scholars' attention. With the continuous research, scholars at home and abroad have a profound understanding of the durability degradation process and deterioration mechanism of bridge structures, and most of them adopt the methods related to accelerated corrosion and have achieved fruitful results [14]. However, the research on the durability of bridge structures is mostly concentrated in the field of general bridges, and relatively little research has been done on new construction materials. Along with the improvement in people's environmental awareness and the requirements of sustainable development, the research on the durability of green bridge structures and accelerated corrosion also needs to be further clarified, to lay a solid theoretical foundation for the promotion and application of green building materials.

Current methods of accelerated corrosion of bridge structures, particularly carbonation and chloride ions under the action of the accelerated corrosion mechanism, are more mature, and more research results based on the acceleration of steel corrosion method have also attracted more and more attention from scholars. However, the electrolyte used in the existing accelerated corrosion process is mostly an aggressive solution, but due to the lack of oxygen supply in the acceleration process, the deterioration mechanism of the reinforcing steel is distorted, and the model of reinforcing steel corrosion is questioned to some extent. There are many models for predicting the service life of bridge structures, but the majority of current research findings are based on a deterministic model, that is the service life under a specific corrosive environment or stress level. There is no denying that the erosion environment in which the bridge structure is situated changes over time, and that the corrosion stress level is also influenced by uncertainties. At the same time, the durability deterioration of the bridge structure is changing. For example, under the action of a single factor, durability is a gradual accumulation of the deterioration process, whereas under the action of multiple factors, the coupling of various factors sometimes slows down the deterioration rate, and sometimes accelerates it, both have a degree of uncertainty, so based on the deterministic model to predict the service life of the bridge, the use of the probabilistic analysis method as a reliability model for life prediction can better reflect the randomness of bridge structure durability deterioration due to various factors.

RETRACTED

Overall, the main problems in the current study are as follows:

1. At present, the research on the durability deterioration mechanism of bridge structures is mostly focused on ordinary silicate bridges, while there is little research based on green building materials, such as recycled bridge structures and magnesium chloride cement bridge structures to accelerate corrosion.
2. In the accelerated corrosion study of bridge structures, especially based on the accelerated corrosion test by electricity, the electrolyte mostly uses aggressive solutions; however, in the accelerated process with the bridge expansion and cracking, the solution is easy to penetrate the cracks resulting in the outflow of rust products, resulting in a certain ambiguity of the durability deterioration process of bridge structures under the effect of accelerated corrosion by electricity.
3. There are many methods for life prediction of bridge structures, and the life prediction model based on stochastic analysis is practical, but the applicability of the probability function in the stochastic analysis method, the calculation of relevant parameters, and the accuracy of the prediction model need to be further determined.
4. The model of the accelerated test prediction method has certain conditions of applicability, so under the premise of improving the accelerated corrosion mechanism, it will be more practical to explore the applicability and accuracy of life prediction of bridge structures based on the reliability analysis model.

RETRACTED

Probabilistic statistical methods can reflect the factors affecting the durability life of bridge structures in a multilevel and all-around way; therefore, this article focuses on the application of probabilistic statistical methods in the durability prediction of bridge structures.

### 3.2. Probabilistic Statistical Methods

Considering the random nature of endurance life data, the correlation between before and after data, and the effectiveness of probabilistic statistics in the face of data and lack of theoretical models, this section will introduce models and methods based on probabilistic statistics used in the problem of predicting the endurance life of bridge structures. These include traditional probabilistic models, such as Bayesian classification models, conditional random field models, etc., and statistical learning theory, which is the basis of machine learning theory [15–17].

Based on the Bayesian formulation, numerous related theories have been developed. In this section, we introduce Bayesian decision theory in statistical pattern recognition and the Bayesian parameter estimation techniques [18] and Bayesian learning techniques used to apply this decision theory in intrusion detection. The statistical decision theory with Bayesian decision-making as the core component is an important foundation of statistical pattern recognition, and the classifier designed based on it has the lowest classification error rate or risk, so it is often used as a criterion to measure the merits of other classifier design methods. When using this method to build a classification model, the following two prerequisites must be met: (1) the probability of the overall of each category of the sample needs to be known; and (2) the number of categories to be classified for decision-making needs to be known. The problem it solves is to determine the class to which the d-dimensional feature vector observed on the feature space *X*=[*x*_1_, *x*_2_, *x*_3_, ..., *x*_*d*_]^*T*^ belongs, so it can be said that the Bayesian decision model-based intrusion detection technique combines both the feature space-based intrusion detection technique and the probabilistic statistics-based intrusion detection technique.

Bayesian decision-making based on the minimum error rate considers the posterior probability *P*(*x*_*i*_ *|* *X*), which *x*_*i*_ denotes the category to which it belongs, and for the binary classification problem, *i* = 1, 2; then, based on the known probability of the overall of each category, this posterior probability is calculated by the Bayesian formula, to determine the category to which it belongs by the probability magnitude. The Bayesian formula is shown as follows:

(1) $$\begin{array}{c} P\left(x_{i}\;|\;X\right)=\frac{P\left(X\;|\;x_{i}\right)P\left(x_{i}\right)}{P\left(X\right)}, \end{array}$$

where *P*(*x*_*i*_) is the prior probability *x*_*i*_ of the class, and *P*(*x*_*i*_ *|* *X*) is the conditional probability of the observation *Xx*_*i*_ under the class, *P*(*X*) is a constant and generally need not be considered. In practice, the prior and conditional probabilities of each class are the premises of Bayesian decision theory. This requires estimation of the probability density function, that is, it requires the use of Bayesian parameter estimation or Bayesian learning to infer the overall distribution given a known sample set *P*(*x*_*i*_ *|* *D*). Although the fuzzy-means clustering method based on soft partition can evaluate the durability of multiple samples to be evaluated and multiple evaluation indicators, due to the problem of data resources, although there are multiple samples, each sample has only two durability. The evaluation index can only show the durability of the component to a certain extent. Unlike traditional parameter estimation, which treats the parameter *θ* to be estimated as a constant, Bayesian parameter estimation treats *θ* as a random variable with a priori distribution. The basic idea is to use the past knowledge of *θ* to give a more realistic estimate of *θ*.

RETRACTED

The Bayesian parameter estimation problem can be described as follows: first, the posterior probability density of the parameter *θ* under known data *Y* is calculated using the following Bayesian formula:

(2) $$\begin{array}{c} P\left(\theta \;|\;Y\right)=\frac{P\left(Y\;|\;\theta \right)P\left(\theta \right)}{P\left(Y\right)}, \end{array}$$

where *P*(*θ*) is the known *θ* prior distribution and is the conditional probability of the sample *Y* under *P*(*Y* *|* *θ*) the parameters *θ*; then, the estimate *θ*=*E*(*θ* *|* *Y*) is calculated according to the *θ* theorem.

Bayesian learning, on the other hand, solves directly for the overall distribution *P*(*x*_*i*_ *|* *Y*) by finding the posterior probability of the parameter *θ*, which is expressed as follows:

(3) $$\begin{array}{c} P\left(x_{i}\;|\;Y\right)=\int P\left(x_{i}\;|\;X\right)P\left(X\;|\;Y\right)\text{d}x_{i}. \end{array}$$

Its learning process is roughly encapsulated as follows: for a fixed, it will completely determine the probability density of *x*; when the sample is observed; as the number of samples increases, the uncertainty of inference on will decrease. The basic theory of statistical pattern recognition is Bayesian decision theory, which has important implications for modelling and designing classifiers for bridge durability life prediction. Because Bayesian parameter estimation and Bayesian learning are both basic probabilistic statistical methods, they can be used in a variety of other durability life prediction models.

RETRACTED

### 3.3. Experimental Design and Analysis of Results

For durability assessment of actual projects, the reliability of the current structural system should be evaluated not only from the system level but also considering the time effect and evaluating the reliability of the system at different moments [19]. The carbonization rate of different parts is different due to various factors, and considering the complexity of the carbonization process, if a single time-varying model is used to deal with the carbonization of the members, the results are too subjective and difficult to match with the specific actual project. Therefore, the Bayesian dynamic carbonation model can be used to make dynamic corrections to the respective carbonation based on the historical inspection data of each part of the real bridge and then calculate the reliability of the structural system based on the corrected carbonation depth (Figure 4).

In the figure *A*_*i*_(*α*, *β*), it indicates the carbonation depth correction value of member *i* at the *α* moment after the moment update; *M*_*i*_(*α*, *β*)=*F*[*A*_i_(*k*, *k* − 1)] is the detection value of member *i* at the moment *β*; *N*_*i*_(*α*, *β*) is the reliability index of member *i* at the moment *α* after the moment *β* update; *N*(*α*, *β*)=*F*[*M*_1_(*α*, *β*),…, *M*_*i*_(*α*, *β*)] is the system reliability index at the moment *α* after the moment *β* update. From the flow chart, it can be seen that the Bayesian dynamic linear model completes the dynamic update correction of the carbonation depth, that is

(4) $$\begin{array}{c} A_{i}\left(\alpha ,\beta \right)=F\left[A\left(k,k-1\right),M\left(i,k\right)\right]. \end{array}$$

The component reliability calculation can be expressed as follows:

(5) $$\begin{array}{c} M_{i}\left(\alpha ,\beta \right)=F\left[A_{i}\left(k,k-1\right)\right]. \end{array}$$

And the differential equivalence recursive algorithm completes the calculation of the component reliability to the system reliability, that is

(6) $$\begin{array}{c} N\left(\alpha ,\beta \right)=F\left[M_{1}\left(\alpha ,\beta \right),\ldots ,M_{i}\left(\alpha ,\beta \right)\right]. \end{array}$$

A top-bearing reinforced concrete box arch bridge with a calculated span of 81 m and a calculated vector height of 13.5 m was selected here. Due to the lack of bridge inspection data, it is difficult to collect the same bridge inspection data for the past years, so the rapid carbonation test of concrete was carried out in the laboratory to replace the actual measured data of the bridge with the test data. The stress state of the members in the test was determined according to the computational model, and Figure 5 shows the comparison of the carbonation depth of each specimen.

RETRACTED

For reinforced concrete arch bridges, the main components can be divided into bridge tunnel system, arch column, main arch ring, etc. The carbonization model of different components is different due to different environments. The speed should be greater than the carbonization speed when there is no stress; while the main arch ring and the columns on the arch are mostly eccentric compression members, under appropriate compressive stress, the concrete is denser, which hinders the entry of carbon dioxide to a certain extent and slows down the carbonization speed. However, if the compressive stress is too large, cracks will occur inside, which may facilitate the entry of carbon dioxide and increase the carbonization rate instead.

The Bayesian dynamic linear model is used to correct and predict the carbonization depth. Taking the updated carbonization depth as the effect and the corresponding protective layer thickness as the resistance, according to the reliability calculation method, the reliability index of the component can be obtained at any time. The reliability index of the bridge system is obtained, and then the differential and equivalent recursive algorithm is used to obtain the reliability index of the bridge system after each update. It can be seen from Figure 6 that with the introduction of their respective test data, the reliability indicators of each component have been revised to different extents. On the one hand, some members become more reliable after the update, and some members become less reliable, which has little effect on the overall correction. It can also be seen from Figure 6 that the reliability changes of different components are different. If we use the reliability of components to evaluate the reliability of the system, not only because of the different selection of components, the evaluation results will also be different, and no matter how you choose, the reliability of components is always greater than the reliability of the system, which is dangerous to a certain extent.

Therefore, when evaluating the durability of bridge structures, it is not only necessary to start from the system level to solve the bias brought by replacing the system with the components, but also to reduce the subjective error by making comprehensive use of previous empirical models and engineering actual measurement data. In the absence of a large amount of statistical information on carbonation, this method can be effectively adapted to each specific project to make a more reliable assessment, and also has an important guiding role for the later maintenance and strengthening.

RETRACTED

The reliability of the system is influenced by many factors, not only the reliability of each member, but also its correlation coefficient, which depends on the limit state equation of each member and is influenced by the thickness of the protective layer and the depth of carbonation. The influence of the reliability of each member on the reliability of the system is studied to determine the sensitivity of each member to the system and to provide guidance for the design and testing of reinforcement. The material fracture prediction is closely related to the material type, chemical composition, and manufacturing process, and its magnitude is the key factor determining the fatigue crack propagation characteristics of the structural details of the steel bridge deck. The fracture parameter values of different steels are quite different and show significant random characteristics due to the influence of the inhomogeneity of the material microstructure. The thickness of the protective layer of the members directly affects the reliability of the members. The thickness of the protective layer of each member is changed from 24 mm to 36 mm, and the thickness of the protective layer of one member is changed each time, and the reliability index is calculated on the 30th day after the fourth update. *β* = 3.24.

From Figure 7(a), it can be seen that when the thickness of the protective layer is 30 mm, the change in the thickness of the protective layer of the bridge deck has the greatest influence on the reliability of the system and increasing the thickness of the protective layer of the bridge deck within a certain range can improve the reliability of the system, while increasing the thickness of the protective layer of the arch ring and column, the reliability of the system is not obvious; if the thickness of the protective layer of the bridge deck is reduced, the reliability of the system will be reduced immediately, while the thickness of the protective layer of the arch ring and column will be reduced by a certain amount before the reliability of the system decreases sharply. After a certain amount, the reliability of the system will drop sharply. When the thickness of the protective layer remains unchanged, the reliability index of the bridge deck is the lowest, and the reliability change of the bridge deck has the greatest influence on the reliability of the system, and the component with the greatest influence on the reliability of the system or the component with the lowest reliability, in order to further investigate the change law, makes the change of the reliability caused by the thickness of the respective protective layer and the change of the reliability of the corresponding system, as shown in Figures 7(b)–7(d), where Figures 7(b) and 7(c) make the auxiliary line *y* = . From the graph, it can be seen that the system reliability index is always lower than the reliability index of each member, according to the analysis of Figures 7(c) and 7(d), when the thickness of the protection layer of column or arch ring increases, the reliability index of the bridge deck remains unchanged, and the lowest reliability index is the bridge deck; therefore, when the thickness of the protection layer of column and arch ring increases, the system reliability can only be infinitely close to that of the bridge deck. The reliability of the system can only be infinitely close to the reliability index of the bridge deck; while the reliability of the bridge deck is still the lowest when the thickness of the protective layer of the column or the arch ring is reduced, and the change of the system reliability is not much when the thickness of the protective layer is reduced to the reliability index lower than that of the bridge deck, the system reliability index will be reduced with the reliability of the arch ring or the column; from Figure 7(d), it can be seen that for the bridge deck, the reliability is lower than that of the arch ring and the column because the reliability is lower than that of the bridge deck. Therefore, the change of protection layer thickness directly affects the system reliability index, and when the protection thickness increases to the extent that the reliability index of the deck plate is larger than that of the column, the change in system reliability gradually becomes smaller and lower than that of the column, which has the lowest member reliability at this time.

RETRACTED

It can be seen from Figures 8(a) and 8(b) that when there is arch or column maintenance, although the member reliability can be temporarily stopped, the improvement in the system is not large, because at this time the system has the greatest impact on the components for the lowest reliability of the bridge deck, so the arch and column maintenance on the system is not much, and from Figure 8(c), it can be seen that when there is bridge deck maintenance, the system reliability decreases significantly slower, indicating that the maintenance of the bridge deck plate has a certain slowing effect on the system, but the system reliability is still decreasing at this time, which also shows that the members are only part of the system, and the influence of a single member on the system is limited. The maintenance of the deck slab has a more obvious improvement on the system's durability. According to the calculation results, the system reliability index is improved by 2.55% after the maintenance of the deck slab, while the arch ring and column are improved by 0.15% and 0.29%, respectively, after the maintenance. Therefore, when maintaining the bridge, the deck plate should be considered first, and if the reliability is no longer the lowest after the deck plate maintenance, the member with the lowest reliability at that moment should be considered for maintenance if maintenance is still needed.

Because the maintenance of the bridge deck plate has a more obvious impact on the system's reliability, the reliability index comparison is calculated separately when the bridge deck is maintained at different carbonation times, as shown in the experiment above, to investigate the impact of the maintenance time point on the change in reliability. The a priori model is modified by combining the testing data, based on the Bayesian dynamic linear model, so that the initial general a priori model can continuously incorporate the individual characteristics of the structure and the results are closer to the actual conditions. According to the analysis, the reliability index change curve shifts to the right after maintenance, and because the distance shifted is the same, the final effect of maintenance remains the same as long as maintenance is performed before the failure of the member; however, the system's reliability still decreases when maintenance is performed on a single member, so maintenance of the member before the system's failure does not guarantee.

## 4. Conclusion

The ability of a structure or member to maintain its safety and serviceability within the design life is reflected in its durability. In this article, a combination of experimental analysis, finite element simulation, and theoretical analysis is used to investigate how to incorporate the carbonation model of concrete members with individual characteristics, the durability and reliability of members and their time-varying properties, and the system durability and reliability dyads, all while considering the working conditions of concrete bridges in actual services, such as loading, cracking, and even acid rain erosion. The research looked into dynamic reliability assessment methods. The following are the main conclusions: (1) The carbonation rate of concrete decreases under compressive stress, and the degree of reduction is related to the ratio of compressive stress to ultimate compressive stress; tensile stress facilitates carbonation, and the higher the tensile stress, the faster the carbonation rate. (2) The similarity of the mechanism of action between the carbon dioxide diffusion model and the heat conduction equation is revealed by comparing the two, allowing a finite element model of concrete with cracks to be constructed and the effects of crack width and depth on the carbonation of concrete to be discussed. (3) The a priori model is modified based on the Bayesian dynamic linear model by combining the testing data, so that the initial general a priori model can continuously incorporate the individual characteristics of the structure, and the results are closer to the actual conditions; in the meantime, in response to the finding that the traditional Bayesian dynamic linear model may have a shortage of gradually increasing deviation between the predicted data and the measured data, the a priori model is modified by combining the testing data, so that the initial general idea of stepwise correction of the a priori model and prediction model is proposed, the error correction expression is given, and the idea's effectiveness is tested using the algorithm. (4) By combining the Bayesian dynamic model and the differential equivalence recursive algorithm, a dynamic assessment method for the bridge system's durability is presented, which can dynamically update the structure's durability condition at any time based on inspection data feedback. The algorithm's analysis reveals that there is a risk of replacing system evaluation with component evaluation, and that the components with the lowest reliability in tandem mode have the greatest influence on the system, which should be considered during inspection and maintenance.

RETRACTED

## Figures and Tables

**Figure 1:** Factors affecting the durability life of bridges.

**Figure 2:** The flow of accelerated experimental prediction method.

**Figure 3:** Probabilistic analysis prediction method flow.

**Figure 4:** Flow chart of dynamic reliability assessment.

**Figure 5:** Comparison of the carbonization depth of specimens in each part.

**Figure 6:** Comparison of the reliability of each component of the bridge.

**Figure 7:** Effect of the thickness of the protective layer on the reliability of the system. (a) Protective layer thickness variation (mm), (b) variation of arch ring protection layer thickness (mm), (c) variation of column protective layer thickness (mm), and (d) bridge deck plate protection layer thickness change (mm).

**Figure 8:** Comparison of reliability indicators after the maintenance of different components. (a) Maintenance of bridge deck, (b) maintenance of column, and (c) maintenance of arches.

## Data Availability

The data used to support the findings of this study are available from the author upon request.
